The article "Effect of EtOH/MgCl2 Molar Ratios on the Catalytic Properties of MgCl2-SiO2/TiCl4 Ziegler-Natta Catalyst for Ethylene Polymerization" was published in 2011. Journal: Molecules.

# Effect of EtOH/MgCl_2_ Molar Ratios on the Catalytic Properties of MgCl_2_-SiO_2_/TiCl_4_ Ziegler-Natta Catalyst for Ethylene Polymerization

**DOI:** 10.3390/molecules16108332

**Published:** 2011-09-29

**Authors:** Supanan Patthamasang, Bunjerd Jongsomjit, Piyasan Praserthdam

**Affiliations:** Center of Excellence on Catalysis and Catalytic Reaction Engineering, Department of Chemical Engineering, Faculty of Engineering, Chulalongkorn University, Bangkok 10330, Thailand

**Keywords:** Ziegler-Natta catalyst, silica, MgCl_2_, ethanol, spherical support, morphology, polyethylene

## Abstract

MgCl_2_-SiO_2_/TiCl_4_ Ziegler-Natta catalysts for ethylene polymerization were prepared by impregnation of MgCl_2_ on SiO_2_ in heptane and further treatment with TiCl_4_. MgCl_2_^·^nEtOH adduct solutions were prepared with various EtOH/MgCl_2_ molar ratios for preparation of the MgCl_2_-supported and MgCl_2_-SiO_2_-supported catalysts in order to investigate the effect on polymerization performance of both catalyst systems. The catalytic activities for ethylene polymerization decreased markedly with increased molar ratios of [EtOH]/[MgCl_2_] for the MgCl_2_-supported catalysts, while for the bi-supported catalysts, the activities only decreased slightly. The MgCl_2_-SiO_2_-supported catalyst had relatively constant activity, independent of the [EtOH]/[MgCl_2_] ratio. The lower [EtOH]/[MgCl_2_] in MgCl_2_-supported catalyst exhibited better catalytic activity. However, for the MgCl_2_-SiO_2_-supported catalyst, MgCl_2_ can agglomerate on the SiO_2_ surface at low [EtOH]/[MgCl_2_] thus not being not suitable for TiCl_4_ loading. It was found that the optimized [EtOH]/[MgCl_2_] value for preparation of bi-supported catalysts having high activity and good spherical morphology with little agglomerated MgCl_2_ was 7. Morphological studies indicated that MgCl_2_-SiO_2_-supported catalysts have good morphology with spherical shapes that retain the morphology of SiO_2_. The BET measurement revealed that pore size is the key parameter dictating polymerization activity. The TGA profiles of the bi-supported catalyst also confirmed that it was more stable than the mono-supported catalyst, especially in the ethanol removal region.

## 1. Introduction

Ziegler-Natta (ZN) catalysts have been widely used in polyolefin industrial since the 1950s. The ZN catalyst systems consisted of a Group IV or V metal halide catalyst and Group II or III metal alkyl or alkylhalide cocatalysts. The advantages of supported ZN catalysts are that the morphology of the polymer particles produced can be controlled by varying the morphology of the support and high catalyst activity can be achieved. In the order to meet the requirement of the polyolefin industry, it is important to produce high performance ZN catalysts with good morphology. Among catalyst supports MgCl_2_ is the most widely used one for olefin polymerization Ziegler-Natta catalysts with high performance and high catalytic activity.

The article "Effect of EtOH/MgCl2 Molar Ratios on the Catalytic Properties of MgCl2-SiO2/TiCl4 Ziegler-Natta Catalyst for Ethylene Polymerization" was published in 2011. Journal: Molecules.

Typically, three methods have been used to prepare activated MgCl_2_ supports for ZN catalysts, including physical (ball-milling), and chemical routes (recrystallization and chemical conversion method). Currently, the activation of MgCl_2_ is usually done via the chemical route. The recrystallization of MgCl_2_ in alcoholic hydrocarbon solution is the well-known method to make spherical catalysts [1,2,3]. However, in the synthesis of MgCl_2_ supports via this method it is not easy to obtain compact and good catalyst morphology because it is difficult to control the alcohol content in MgCl_2_-ethanol complexes, which influences the porosity and strength of the catalyst particles and the subsequent polymer-particle morphology due to the replication phenomena [4,5,6,7]. The fragmentation of MgCl_2_-adduct-based catalyst particles is still the important problem during the polymerization, because it can result in undesirable polymer morphology, formation of fines and reactor fouling [8,9].

Silicas are commonly used as supports for many catalysts. They have relatively high surface areas and pore volumes per unit mass. They also have chemically reactive groups on the surface, most of which are within the pore structure. Their particles size and shapes are often controlled to optimize catalyst performance [10,11,12]. However, the disadvantage of SiO_2_-supported ZN catalyst is their low activity [12]. The catalytic activity of SiO_2_-supported Ziegler-Natta catalysts can be improved by addition of MgCl_2_. The bi-supported (MgCl_2_-SiO_2_) ZN catalysts combine the advantages of the controllable morphology of SiO_2_ and the high activity of MgCl_2_ [13,14,15]. Typically, the synthesis of bi-supported ZN catalysts can be done by combination of the MgCl_2_ with SiO_2_, then treating with TiCl_4_ [13,16]. In addition, an electron donor can be used to increase the isotacticity of the bi-supported catalyst for propylene polymerization [17,18]. The impregnation of MgCl_2_ on the SiO_2_ surface is usually used to control the morphology of the bi-supported catalyst. MgCl_2_·nEtOH adduct solution is usually prepared before impregnation on SiO_2_ [19,20]. Forte and Coutinho [5] found that the catalyst preparation conditions apparently affected the chemical composition and morphology of catalyst. The amount of ethanol has a remarkable effect on the preparation of MgCl_2_·nEtOH adduct. Besides, the precipitation of MgCl_2_ and the removal of ethanol are the important parameters to obtain catalyst supports and catalysts with good morphology having spherical catalyst and polymer product shapes.

The article "Effect of EtOH/MgCl2 Molar Ratios on the Catalytic Properties of MgCl2-SiO2/TiCl4 Ziegler-Natta Catalyst for Ethylene Polymerization" was published in 2011. Journal: Molecules.

Presently, it is known that the [EtOH]/[MgCl_2_] ratio is a very important parameter to control the morphology and catalyst performance for MgCl_2_-supported catalysts [4,7]. However, the effect of [EtOH]/[MgCl_2_] ratio on the preparation of MgCl_2_-SiO_2_-supported catalysts is still unknown, even though the deposition of MgCl_2_ on SiO_2_ via MgCl_2_·nEtOH adduct solutions has been used in the preparation of these catalysts. Therefore, in this present study, we have investigated the effect of [EtOH]/[MgCl_2_] ratio on the properties of MgCl_2_-SiO_2_-supported catalysts. The MgCl_2_/TiCl_4_ and MgCl_2_-SiO_2_/TiCl_4_ catalysts were synthesized with various [EtOH]/[MgCl_2_] ratios in the MgCl_2_·nEtOH adduct used for MgCl_2_ impregnation on SiO_2_. The catalytic activity, morphology of catalyst, BET surface area, pore size, pore volume, and thermal properties were investigated and are further discussed in more detail.

## 2. Results and Discussion

### 2.1. Polymerization Activity

MgCl_2_-supported catalysts (M) and MgCl_2_-SiO_2_-supported catalysts (SM) were synthesized with various MgCl_2_·nEtOH adducts having n values ranging from 6 to 10. The supports were then treated with TiCl_4_ to obtain the corresponding mono-supported and bi-supported catalysts. The preparation conditions of both catalyst systems are shown in Table 1. The results show that Ti content of MgCl_2_-supported catalysts was relatively higher than for MgCl_2_-SiO_2_-supported catalysts in the range of 7.00–7.60 and 6.70–7.32 wt%.

**Table 1:** MgCl_2_-supported and MgCl_2_-SiO_2_-supported catalysts preparation conditions.

**MgCl_2_-supported catalyst**					
**Sample**	**EtOH (mL)**	**[EtOH]/[MgCl_2_]**	**TiCl_4_ (mL) ^a^**	**SiO_2_ (g)**	**Ti (wt%)**
M6	11.0	6	18.3	0	7.00
M7	12.9	7	21.4	0	7.34
M8	14.7	8	24.4	0	7.54
M9	16.6	9	27.5	0	7.43
M10	18.0	10	30.0	0	7.60
**MgCl_2_-SiO_2_** **-supported catalyst**					
**Sample**	**EtOH (mL)**	**[EtOH]/[MgCl_2_]**	**TiCl_4_ (mL) ^a^**	**SiO_2_ (g)**	**Ti (wt%)**
SM6	11.0	6	18.3	6	6.93
SM7	12.9	7	21.4	6	6.80
SM8	14.7	8	24.4	6	6.77
SM9	16.6	9	27.5	6	6.70
SM10	18.0	10	30.0	6	7.32

Note: ^a^ The desired amount of TiCl_4_ using for removing of EtOH from MgCl_2_ adduct calculated by [EtOH]/[TiCl_4_] = 1.13.

Ethylene polymerization was performed using both catalyst systems. Figure 1 shows that the catalytic activities of the mono-supported (M) catalysts were markedly decreased with increased [EtOH]/[MgCl_2_] ratios of 6 to 10, whereas the activities were only slightly decreased for the bi-supported (SM) catalysts for the identical [EtOH]/[MgCl_2_] ratios. It should be mentioned that the MgCl_2_-SiO_2_-supported catalysts usually have lower activity than MgCl_2_-supported catalysts because of the high number of silanol groups on the SiO_2_ surface [21,22]. However, based on this study at [EtOH]/[MgCl_2_] ratios of 9 and 10, the bi-supported catalysts showed higher activity than the mono-supported catalyst, as seen in Figure 1 for SM9 and SM10 compared to M9 and M10.

The article "Effect of EtOH/MgCl2 Molar Ratios on the Catalytic Properties of MgCl2-SiO2/TiCl4 Ziegler-Natta Catalyst for Ethylene Polymerization" was published in 2011. Journal: Molecules.

In the case of MgCl_2_-supported catalysts, [EtOH]/[MgCl_2_] ratio is an important parameter and this catalyst system prefers lower [EtOH]/[MgCl_2_] during support preparation to give better catalytic activity and performance [6,23]. An excess amount of EtOH in the support could react with TiCl_4_, and produce inactive species like Ti alkoxide [24]. In contrast, the bi-supported catalysts showed the interesting result that the activity was relatively independent of the [EtOH]/MgCl_2_] ratio. This indicates that the SiO_2_ probably prevents the Ti active species from reacting further with ethanol.

**Figure 1:** Effect of [Ethanol]/[MgCl_2_] on catalytic activity and relative activity of MgCl_2_-SiO_2_-supported catalyst (SM) and MgCl_2_-supported catalyst (M). Ethylene polymerization condition: temperature = 80 °C; catalyst loading = 10 mg; [A1]/[Ti] = 100; ethylene consumption = 18 mmol.

### 2.2. Effect of [EtOH]/[MgCl_2_] on Morphology of bi-Supported Catalysts

Scanning electron microscopy (SEM) measurements revealed that the spherical morphology of SiO_2_ is retained by the catalyst. In this study, MgCl_2_-ethanol solutions with [EtOH]/[MgCl_2_] ratios of 6, 7, 8, 9 and 10 were used to prepare catalysts. The minimum amount of ethanol to completely dissolve the MgCl_2_ and for impregnation of the SiO_2_ was 6 under the experimental conditions used. The viscosity of the adduct solution increases with decreasing amounts of ethanol, hence being more difficult with impregnation at [EtOH]/[MgCl_2_] ratios <6.

The external morphology of the SiO_2_ and the MgCl_2_-SiO_2_-supported catalysts was seen by SEM (Figure 2). The SEM micrographs of the bi-supported catalysts shown in Figure 2 indicating that the catalyst particles retain the shape of the SiO_2_ precursor particles. However, the SEM images also revealed that some breakage of particles occurred. The surfaces of bi-supported catalysts were rough, with some agglomeration of MgCl_2_, as shown in the SEM images. Figure 2(c-d) show images of SM6 catalyst prepared with [EtOH]/[MgCl_2_] = 6. It was found that the MgCl_2_ was crystallized on the surface of bi-supported catalyst. The concentration of MgCl_2_ in ethanol is one of important factors in the impregnation process. As known, if the adduct solution prepared has a high concentration of MgCl_2_, it will exhibit high viscosity that will make it unable to disperse into the pores of SiO_2_ and resulting in agglomeration on the external surface. 

The article "Effect of EtOH/MgCl2 Molar Ratios on the Catalytic Properties of MgCl2-SiO2/TiCl4 Ziegler-Natta Catalyst for Ethylene Polymerization" was published in 2011. Journal: Molecules.

**Figure 2:** SEM images of **(a)** and **(b)** SiO_2_ and MgCl_2_-SiO_2_-supported catalysts prepared with various of [EtOH]/[MgCl_2_] ratios; **(c)** and **(d)** SM6, **(e)** and **(f)** SM7, **(g)** and **(h)** SM8, **(i)** and **(j)** SM9, **(k)** and **(l)** SM10.

However, upon drying precipitation of MgCl_2_ on the external surface of the SiO_2_ was observed as an external rough surface for SM6. On the other hand, at higher [EtOH]/[MgCl_2_] values of 7 and 8, the catalyst surface became smooth and very little agglomeration of MgCl_2_ on the catalyst surface was observed, as shown in Figure 2(e-f) and (g-h). However, at [EtOH]/[MgCl_2_] values of 9 and 10, cracking on the bi-supported catalyst surfaces was observed, as shown in Figure 2(i-j) and (k-l). This may be due to brittle films of impregnated MgCl_2_ caused by the high ethanol content. Therefore, the effect of [EtOH]/[MgCl_2_] on morphology structure of MgCl_2_ deposited on the SiO_2_ surface is similar to that on the MgCl_2_-supported catalyst in terms of producing loose and breakable MgCl_2_ structures with high ethanol content [1].

Therefore, MgCl_2_-SiO_2_-supported catalyst requires an optimal [EtOH]/[MgCl_2_] ratio due to the viscosity limitation that can affect the impregnation and dispersion of MgCl_2_ on the SiO_2_ surface. MgCl_2_ can agglomerate on the SiO_2_ surface with low [EtOH]/[MgCl_2_] and it is not suitable for loading TiCl_4_ on the MgCl_2_-SiO_2_-support. The optimized [EtOH]/[MgCl_2_] value for preparing bi-supported catalysts having high activity and good spherical morphology with little agglomeration of MgCl_2_ is 7 under these experimental conditions.

### 2.3. Determination of Surface Area

Surface areas of mono- and bi-supported catalysts were determined by the BET method. The results are listed in Table 2. The bi-supported catalysts exhibited much higher surface areas than the mono-supported catalysts prepared under similar [EtOH]/[MgCl_2_] ratios due to the high surface area of SiO_2_ in the bi-supported catalyst. The bi-supported catalysts containing different [EtOH]/[MgCl_2_] values of MgCl_2_ adduct exhibit similar surface area of 414–471 m^2^/g, pore size of 44.6–52.5 Å and pore volume of 0.46–0.60 cm^3^/g. Therefore, the relatively constant bi-supported catalyst structure is the reason for the relatively constant catalytic activity. The BET measurements of mono-supported catalyst showed that the surface area, pore size and pore volume of the catalysts depended on the [EtOH]/[MgCl_2_] ratios (as seen for M6 and M10 in Table 2). The results show that M6 prepared with a low [EtOH]/[MgCl_2_] value exhibited much larger pores than those of M10 prepared with a higher [EtOH]/[MgCl_2_] value. The larger pores size may be responsible for the higher catalytic activity of M6 compared to M10.

The article "Effect of EtOH/MgCl2 Molar Ratios on the Catalytic Properties of MgCl2-SiO2/TiCl4 Ziegler-Natta Catalyst for Ethylene Polymerization" was published in 2011. Journal: Molecules.

**Table 2:** BET surface area measurement of MgCl_2_-supported catalysts and MgCl_2_-SiO_2_-supported catalysts.

Catalyst name	BET surface area(m^2^/g)	Pore size (diameter) (Å)	Pore volume (cm^3^/g)
SiO_2_ (SYLOPOL 2229)	489	97.22	1.60
M6	187	88.00	0.53
M10	366	39.30	0.36
SM6	419	49.60	0.51
SM7	455	52.50	0.60
SM8	450	50.40	0.57
SM9	471	46.40	0.55
SM10	414	44.60	0.46

### 2.4. Thermal Analysis

Figure 3 shows TGA profiles of MgCl_2_-supported catalysts and MgCl_2_-SiO_2_-supported catalyst. It indicates that bi-supported catalysts exhibited the similar TGA profiles as SiO_2_, with a relative decrease the weight loss with temperature after 200 °C. The bi-supported catalysts retained over 80% of their mass when heated to 500 °C (mass loss ≤ 20%) while the mono-supported catalyst lost about 50% of their mass for the same thermal treatment. TGA profiles show that the mono-supported catalysts have significant mass losses in the range of 70 to 190 °C (30 to 40%). The ethanol content in MgCl_2_-supported catalyst was more than the MgCl_2_-SiO_2_-supported catalyst. This was due to the preparation procedures between MgCl_2_ and MgCl_2_-SiO_2_ supports were different in the weight ratio of support/EtOH.

**Figure 3:** TGA profiles of MgCl_2_-supported catalysts (M) and MgCl_2_-SiO_2_-supported catalysts (SM).

EtOH and moisture escaped from surface and catalyst particles in this temperature range. The mono-supported catalysts have a maximum weight loss from 150–190 °C in M6 catalyst and 70–130 °C in M10 catalyst, indicating that at a higher [EtOH]/[MgCl_2_] value as 10, ethanol groups were removed easily from the catalysts because of the loose structure of M10 produced with a high content of ethanol [1]. This may be the reason why the decrease of weight loss of M10 was sharper and started earlier than those of M6. On the other hand, the bi-supported catalysts show only a slight decrease of weight loss profile. The results also show that at 200 °C, the bi-supported catalysts have an average weight of 90% corresponding to a weight loss of 10%, whereas the mono-supported catalysts exhibited average weights of 68%, corresponding to a weight loss of 33%.

## 3. Experimental

### 3.1. Chemicals

Anhydrous MgCl_2_ (Toho) was used as received. SiO_2_ (SYLOPOL 2229, received from Grace Davison having particle size of 40–50 mm and surface area of 270 m^2^/g) was calcined at 600 °C for 6 h. Ethanol (Merck Ltd.) was dried with 4 Å molecular sieves. TiCl_4_ (Merck Ltd.) was used as received. Heptane and toluene (Merck Ltd.) were purified by distillation with Na metal/benzophenonone in an atmosphere of high purity Ar to remove residual traces of moisture and oxygen. Ultra high purity (UHP) argon (99.999%) was purchased from Thai Industrial Gas Co., Ltd. and was further purified by passing through 3 Å molecular sieves, BASF catalyst R3-11G, NaOH and phosphorus pentoxide (P_2_O_5_) to remove traces of oxygen and moisture. Polymerization grade ethylene and triethylaluminum (TEA) were donated by PTT Public Co., Ltd. Standard Schlenk techniques and high purity argon were used for the handling of all compounds.

The article "Effect of EtOH/MgCl2 Molar Ratios on the Catalytic Properties of MgCl2-SiO2/TiCl4 Ziegler-Natta Catalyst for Ethylene Polymerization" was published in 2011. Journal: Molecules.

### 3.2. Catalyst Preparations

#### 3.2.1. MgCl_2_-Supported Catalyst Preparation

A 300 mL 3-necked round bottom flask equipped with mechanical stirrer, Ar inlet and outlet lines and cooling system were used in the preparation. Anhydrous MgCl_2_ (3.0 g) was suspended in heptane (20 mL), and then the desired amount of ethanol was added to the slurry with a syringe under Ar. The mixture was heated to 80 °C and stirred until MgCl_2_ was completely dissolved. Then, the MgCl_2_ adduct solution was cooled to −20 °C and the desired amount of TiCl_4_ was added dropwise at a rate of 25 mL/h. The temperature was slowly increased to 80 °C and kept there for 1 h. The solid was washed with heptane (50 mL) for 3 times. TiCl_4_ (18 mL) and heptane (18 mL) was added into the mixture to activate an intermediate at 95 °C for 1 h. The supernatant was removed, and the solid catalyst was washed several times with heptane. The final catalysts were dried in a vacuum at room temperature and kept under Ar atmosphere.

#### 3.2.2. MgCl_2_-SiO_2_-Supported Catalyst Preparation

The 300 mL 3-necked round bottom flask equipped with mechanical stirrer, Ar inlet and outlet line and cooling system were used in the preparation. Anhydrous MgCl_2_ (3.0 g) was suspended in heptane (20 mL), and then the desired amount of ethanol was added to the slurry under a stream of Ar. The mixture was heated to 80 °C and stirred until MgCl_2_ was completely dissolved. Then, SiO_2_ (6.0 g) in heptane (40 mL) was transferred to reactor using a Teflon tube while stirred. The slurry mixture was stirred for 1 h at 80 °C. The impregnated MgCl_2_ adduct/SiO_2_ was cooled to room temperature with continuous stirring. The solid was washed with toluene (50 mL) two times and heptane (50 mL) two times to remove the alcohol. Heptane (60 mL) was added into 3-necked flask, and then, the slurry was cooled to −20 °C. Consequently, TiCl_4_ was added dropwise at a rate of 25 mL/h. The temperature was slowly increased to 80 °C and kept there for 1 h. The solid was washed with heptane (50 mL) 3 times. TiCl_4_ (18 mL) and heptane (18 mL) were added into the mixture to activate an intermediate at 95 °C for 1 h. The supernatant was removed, and the solid catalyst was washed with heptane several times. The resultant bi-supported catalysts were dried in vacuum at room temperature and kept under Ar atmosphere. 

The article "Effect of EtOH/MgCl2 Molar Ratios on the Catalytic Properties of MgCl2-SiO2/TiCl4 Ziegler-Natta Catalyst for Ethylene Polymerization" was published in 2011. Journal: Molecules.

The nomenclature used is as follows:

MI refers to the MgCl_2_-supported ZN catalyst with [EtOH]/[MgCl_2_] ratio of I.
SMI refer to the MgCl_2_-SiO_2_-supported ZN catalyst with [EtOH]/[MgCl_2_] ratio of I.

### 3.3. Ethylene Polymerization

A 100 mL stainless steel autoclave equipped with a magnetic agitator was used under semi-batch operation. Ethylene polymerization was conducted using catalyst powder (0.01 g), hexane (30 mL), triethylaluminum, Al/Ti = 100, and polymerization at 80 °C and 50 psia total pressure with continuous feeding of ethylene. The reaction was stopped when 18 mmol of ethylene monomer was consumed by venting the monomer and quenching with HCl/methanol. The obtained polymer was washed several times with methanol, filtered and dried under vacuum at 60 °C for 6 h. Due to the fixed ethylene consumption (18 mmol), the polymerization time was defined as the time that all ethylene monomer was completely consumed equivalent pressure drop of 42 kPa (6 psi). The polymerization time was recorded to calculate the catalytic activity. 

### 3.4. Characterization

Morphological study of MgCl_2_-SiO_2_-supported catalyst was investigated using scanning electron microscopy (SEM, JEOL mode JSM-6400). Measurement of BET surface area, pore volume and pore size diameter of catalysts were determined by N_2_ physisorption and Kelvin condensation using a Micromeritics ASAP 2000 automated system. Thermogravimetric analysis (TGA) was performed using a TA Instruments SDT Q 600 analyzer with temperature ramping from 40 to 500 °C at 10 °C/min. The carrier gas was N_2_ (UHP). The Ti content in catalysts was determined by inductively coupled plasma spectroscopy (ICP) using the Perkin-Elmer Plasma 1000 system.

## 4. Conclusions

Mono-supported catalysts (MgCl_2_/TiCl_4_) and bi-supported catalysts (MgCl_2_-SiO_2_/TiCl_4_) were synthesized using various [EtOH]/[MgCl_2_] ratios. The bi-supported catalysts had relatively constant activities with increasing the ethanol/MgCl_2_ ratios due to prevention of the Ti active species from further reaction with ethanol. Activities of the bi-supported catalysts were slightly reduced from the maximum activity, but those of the mono-supported catalyst showed a remarkable reduction with increasing [EtOH]/[MgCl_2_] ratio. The bi-supported catalysts retain the morphology of the SiO_2_ precursor to the catalyst, with spherical shapes. The [EtOH]/[MgCl_2_] ratios affect the bi-supported catalyst morphology in terms of the impregnated film of MgCl_2_ on SiO_2_ surface. Even though lower [EtOH]/[MgCl_2_] ratios in MgCl_2_-supported ZN catalyst give better catalytic activity and particle morphology, the MgCl_2_-SiO_2_-supported ZN catalysts requires moderate [EtOH]/[MgCl_2_] ratios due to their viscosity limitation that can affect impregnation and dispersion of MgCl_2_ on the SiO_2_ surface. In addition, MgCl_2_ can agglomerate on the SiO_2_ surface at low [EtOH]/[MgCl_2_] ratios and this is not suitable for TiCl_4_ loading on the MgCl_2_-SiO_2_-support. The optimized [EtOH]/[MgCl_2_] value for preparing bi-supported catalysts with high activity and good spherical morphology with little agglomeration of MgCl_2_ is 7. The bi-supported catalyst has high specific surface area and porosity without any relationship between activity of catalyst and surface area. Additional, thermal properties show that TGA profiles of the bi-supported catalysts are more stable than the mono-supported catalysts, especially in the region of ethanol and moisture removal.
